The article "Specific clones of Trichomonas tenax are associated with periodontitis" was retracted in 2024. Reasons: errors in the text; lack of ethics approval or compliance; a conflict of interest; concerns about the data.

# Specific clones of *Trichomonas tenax* are associated with periodontitis

**DOI:** 10.1371/journal.pone.0213338

**Published:** 2019-03-11

**Authors:** Sarah Benabdelkader, Julien Andreani, Alexis Gillet, Elodie Terrer, Marion Pignoly, Herve Chaudet, Gerard Aboudharam, Bernard La Scola

**Affiliations:** 1 Aix-Marseille Université UM63, Institut de Recherche pour le Développement IRD, Assistance Publique–Hôpitaux de Marseille (AP-HM), Microbes, Evolution, Phylogeny and Infection (MEΦI), Institut Hospitalo-Universitaire (IHU) - Méditerranée Infection, Marseille, France; 2 UFR Odontologie, Aix-Marseille Université, Marseille, France; Klinikum der Johann Wolfgang Goethe-Universitat Frankfurt Klinik fur Nuklearmedizin, GERMANY

## Abstract

*Trichomonas tenax*, an anaerobic protist difficult to cultivate with an unreliable molecular identification, has been suspected of involvement in periodontitis, a multifactorial inflammatory dental disease affecting the soft tissue and bone of periodontium. A cohort of 106 periodontitis patients classified by stages of severity and 85 healthy adult control patients was constituted. An efficient culture protocol, a new identification tool by real-time qPCR of *T*. *tenax* and a Multi-Locus Sequence Typing system (MLST) based on *T*. *tenax* NIH4 reference strain were created. Fifty-three strains of *Trichomonas* sp. were obtained from periodontal samples. 37/106 (34.90%) *T*. *tenax* from patients with periodontitis and 16/85 (18.80%°) *T*. *tenax* from control patients were detected by culture (p = 0.018). Sixty of the 191 samples were tested positive for *T*. *tenax* by qPCR, 24/85 (28%) controls and 36/106 (34%) periodontitis patients (p = 0.089). By combining both results, 45/106 (42.5%) patients were positive by culture and/or PCR, as compared to 24/85 (28.2%) controls (p = 0.042). A link was established between the carriage in patients of *Trichomonas tenax* and the severity of the disease. Genotyping demonstrates the presence of strain diversity with three major different clusters and a relation between disease strains and the periodontitis severity (p<0.05). More frequently detected in periodontal cases, *T*. *tenax* is likely to be related to the onset or/and evolution of periodontal diseases.

## Introduction

Periodontal disease is a widespread oral disease affecting adults and younger people, characterized by an inflammatory reaction that affects periodontium tissue [1]. A new classification published in 2018 based on description (localized or generalized), severity and complexity of management divides periodontitis into 4 stages, including initial periodontitis (I), moderate periodontitis (II), severe periodontitis with potential for additional tooth loss (III) and advanced periodontitis with extensive tooth loss and potential for loss of dentition (IV) [2]. According to this classification, periodontitis is also graded in 3 levels estimated with direct or indirect evidence of progression rate: slow (A), moderate (B) and rapid (C). Periodontal disease is characterized by receding gums, alveolar bone destruction, loss of dental junctions associated with the apparition of periodontal pockets, and in some forms, dental calculus deposits. This promotes the establishment of an anaerobic microenvironment that allows the growth of anaerobic microorganisms [3]. The immunological process initiates the migration of microorganisms into tissues and disrupts the immune response, causing the periodontium to resorb [4,5]. Some host risk factors have now been clearly identified, including smoking [6] and diabetes mellitus [7], but other genetic factors require further study [8].

The article "Specific clones of Trichomonas tenax are associated with periodontitis" was retracted in 2024. Reasons: errors in the text; lack of ethics approval or compliance; a conflict of interest; concerns about the data.

The human oral cavity contains an abundant and polymorphic microbiota. A set of bacterial complexes living in subgingival plaque has been identified by Socransky et al; with the initial establishment of Streptococcus spp. and their disappearance, multiple complexes defined by green purple or yellow colors have been described but only the orange and red complexes have been suspected of being associated with the development of periodontitis [3]. Metagenomic studies confirm the association of certain bacterial species found in the orange complex, such as *Prevotella intermedia*, *Prevotella nigrescens* and *Fusobacterium nucleatum* [9,10]. But also the strong association of the disease with the three bacteria described in the red complex: *Pophyromonas gingivalis*, *Tannerella forsythia* and *Treponema denticola* are also found in the periodontal pockets by metagenomic recent studies[11,12] and new species involved have recently been identified [13]. Nevertheless, the “red complex” theory remains debatable due to its isolation in healthy controls (30%, 3/10) [14]. An increase in lytic phages in pathological situations also disturbs the periodontal-associated bacteria present [15]. Similarly, meta-transcriptomics analysis showed that the transcription of bacterial virulence factors increased in patients with periodontitis compared to healthy individuals [16]. Viral etiology has also been suggested as being involved in the development of periodontitis, and different viruses have been involved including Herpesviruses (HSV-1), Cytomegalovirus (CMV) and Epstein-Barr virus (EBV) [17].

Since the 1980s, the implication of eukaryotes in periodontal disease has also been proposed [18], such as the protists *Trichomonas tenax* and *Entamoeba gingivalis* [19–21] and yeasts, such as *Candida* sp. [22]. However, until now, studies focusing on the association between protists and periodontal disease did not use groups of healthy controls to differentiate between abnormal proliferation and natural colonization [20]. Like its neighboring species, *Trichomonas vaginalis*, the vaginitis-inducing pathogen, *T*. *tenax* belongs to the Parabasalia phylum and to the *Trichomonadidae* family [23]. *Trichomonas tenax* can ingest bacteria and various particles by phagocytosis necessary for their development[24]. Initially identified as an harmless commensal [18], then known as a zoonotic parasite [25], this microorganism was detected in the periodontal pockets using mostly optical microscopy [26,27], with an occurrence in patients ranging from 0 to 94.1% depending on the country and the detection procedure [21]. *T*. *tenax* has occasionally been isolated in cases of the salivary glands, lymph nodes or respiratory tract infections [28][29][30]. Recently, *T*. *tenax* was found to be significantly more prevalent in patients with Down syndrome combined with periodontal lesions (14/52), using 18S rRNA gene PCR in comparison to control patients (5/52), with a non-significant difference in plaque indexes between the two groups [31].

The article "Specific clones of Trichomonas tenax are associated with periodontitis" was retracted in 2024. Reasons: errors in the text; lack of ethics approval or compliance; a conflict of interest; concerns about the data.

In this cohort study, we sought to estimate the prevalence of *T*. *tenax* and establish a potential link with the periodontitis severity. We investigated the presence of *T*. *tenax* in periodontitis as compared to the healthy controls using culture and quantitative molecular detection systems. We also used a genome-based system of strain typing to investigate the possibility that a clone or a group of clones of *T*. *tenax* with particular pathogenicity are involved in periodontitis.

## Materials and methods

### Clinical sample collection and treatment

This study was carried out in accordance with the recommendations and approved by the clinical research ethics committee, IFR 48, Aix-Marseille University (protocol N° 2016–011). All subjects gave a written informed consent in accordance with the Declaration of Helsinki. One hundred and ninety-one adults were prospectively enrolled in this cohort, 106 adult patients with periodontitis and 85 healthy adult control patients, (**S1 Table**). The study took place in the Odontology Department of the Hospital La Timone, Marseille, France, between January 2015 and June 2016. The 106 patients with periodontitis could be separated in three classes of severity: 19 patients with mild periodontitis (M), 27 with moderate periodontitis (Mo) and 60 with severe periodontitis (S) according to a previously reported scale using various criteria evaluation: size of the probing depth and the attachment loss for each patient [32]. Smoking status was also collected (**S1 Table)**. Subgingival dental plaque samples were collected from multiple periodontal pocket and combined into a single tube per patient for the group test and the same method was used for healthy gingival sites in the control group. The sample was collected using a sterile Gracey curette (HuFriedy, Rotterdam, Netherlands) and transported into 1 mL of transport medium (C-top Ae-Ana, Eurobio, France). The samples were analyzed according to the detailed protocol in **Fig 1**.

The article "Specific clones of Trichomonas tenax are associated with periodontitis" was retracted in 2024. Reasons: errors in the text; lack of ethics approval or compliance; a conflict of interest; concerns about the data.

**Fig 1:** Schematic protocol for *Trichomonas tenax* studies.

### Isolation of *Trichomonas tenax*

Twelve-and-a-half cm^2^ vented flasks (Corning, NY, USA) containing 10 mL of liquid ATCC: 1171 TYGM-9 medium without rice starch were used to inoculate 250 μL of the clinical samples. The medium was supplemented with 100 Units/mL of Penicillin-Streptomycin Gibco (ThermoFisher, MA, USA) and 20 μg/mL Voriconazole (Sigma-Aldrich, United-States) to retard the bacterial and fungi growth that may interfere with the *T*. *tenax* development. Flasks were then incubated under anaerobic conditions using Anaerogen generators (ThermoFisher, MA, USA) at 35°C. Growth was observed by optical microscopy examination. For the strains cryopreservation, cultures were centrifuged at 720 x g for 10 minutes. The final pellet was suspended in 1 mL of TYGM9 medium containing 1% of di-methyl-sulfoxide (DMSO) and placed in a Nunc cryotube, maintained at -80°C for between 15 and 20 hours before being placed inside a -150°C freezer.

### Molecular identification and typing of isolates

#### Primer design

Based on the analysis of Malik *et al*.[33], we designed specific primers in the 3,048 bp sequence of the RNA polymerase II *rpb1* gene available on the NCBI website (accession number: HM016234.1 for *T*. *tenax* strain NIH4). Primers were designed using Primer-BLAST (https://www.ncbi.nlm.nih.gov/tools/primer-blast/) with standard parameters (**Fig 1F**).

#### Genome sequencing of *Trichomonas tenax*

Briefly, 15 vented Corning 75cm^2^ (NY, USA) flasks containing LYI medium of *T*. *tenax* NIH4 reference strain (ATCC number 30207) were pelleted at 2000 g for 15 minutes, rinsed twice with the same centrifugation parameters in Page’s amoeba Saline before final re-suspension in 1 mL of phosphate buffered saline. Concentrated cells were placed at -80°C before DNA extraction and sequencing. Genomic DNA was sequenced using the Illumina MiSeq (Illumina, Inc, San Diego CA 92121, USA).

The gDNA was quantified by a Qubit assay (Life technologies, Carlsbad, CA, USA) to 6.3 ng/μL and dilution was performed requiring 1 ng of DNA as input. The genomic DNA was fragmented and tagged. Limited cycles of PCR amplification completed the tag adapters and introduce dual-index barcodes. After purification on AMPure beads (Life Technologies, Carlsbad, CA, USA), libraries were then normalized on specific beads according to the Nextera XT protocol (Illumina). Normalized libraries were pooled into a single sequencing library, the MiSeq. The pooled single strand library was loaded onto the reagent cartridge and then onto the instrument along with the flow cell. Automated cluster generation and paired-end sequencing with dual index reads was performed in a single 39-hour, 2x251- base pair run (bp). Total information of 10.5 Gb was obtained from a cluster density of 1,288,000 per mm^2^ with 86.3% (20,305,000 clusters) of the clusters passing quality control filters. Within this pooled run, the index representation of *T*. *tenax* was determined to 39.43%. The 8,005,980 paired end reads were filtered according to the read qualities.

The article "Specific clones of Trichomonas tenax are associated with periodontitis" was retracted in 2024. Reasons: errors in the text; lack of ethics approval or compliance; a conflict of interest; concerns about the data.

#### Multilocus sequence typing

The reads obtained were assembled using the CLC Genomics Workbench. Protein sequences were predicted using the Prodigal platform [34] and analysis. A local Blastp on the predicted proteins was performed on NCBI Blast (Basic Local Alignment Search Tool) against non-redundant protein sequences (nr) database using the standard parameters. The *T*. *tenax* NIH4 genome sequence was deposited on the EMBL-EBI website (Bioproject: PRJEB22701 and whole contigs under accession numbers OCTD01000001-OCTD01004161). Seven single-family household genes were selected ranging in length from 450 to 500 bp **(Table 1)** based on MLST designed for *Trichomonas vaginalis* [35].

**Table 1:** Primers used for multilocus sequence typing genes of *Trichomonas tenax*.

Genes	Forward	Reverse	Sequence length (bp)	No of alleles
Alanyl tRNA synthetase (ALTS)	5’-CCGTCCAGGATGGTGTCTTC-3’	5’-GTAACATCGAATGGCTGGCAC-3’	514	5
DNA mismatch repair protein (DMRP)	5’-ATTGGACAATGGAACCAGTCA-3’	5’-TGACCATATTTCGCACCACG-3’	516	5
Serine hydromethyltransferase (SHMT)	5’-GAGCGATGGAGGACATTTGAC-3’	5’-TTTGGTGAAGATGAGGACCACC-3’	452	4
Mannose-6-phosphate isomerase (M6PI)	5’-AGGTGTTGCAGAGGAGTTGG-3’	5’-TGCTATTTCGTTTGCAGGAACA-3’	421	7
Glutamine amidotransferase class-I (GAT1)	5’-TCTGTTGCACAAGGTCTCAA-3’	5’-TTGTGTAGCCGCCGTATTTG-3’	424	3
Histidyl tRNA synthetase (HIST)	5’-CGTCTCCATCGACACACCAG-3’	5’-TCCATCTCGTCGAGGACCTT-3’	658	8
Cysteinyl tRNA synthetase (CYST)	5’-GCCCGACTGTTTACTCGACA-3’	5’-CGAAGATCGATACCACCGCA-3’	657	0

Single standard PCRs were performed to allow DNA amplification of each selected gene. Primer hybridization was conducted at 59°C and amplified products were sequenced as described previously [36]. Sequences were corrected and assembled using the ChromasPro software version 1.71 (Technelysium, Australia). Obtained sequences were aligned using MUSCLE tool in the Molecular Evolutionary Genetics Analysis software (MEGA) version 7.0.18 (Pennsylvania State University, United-States) and, finally, phylogenetic trees were generated using the maximum-likelihood (ML) method within FastTree version 2.0 [37]. MLST nucleotide sequences data are available in the EMBL-EBI database under accession numbers LT934459 to LT934497.

The article "Specific clones of Trichomonas tenax are associated with periodontitis" was retracted in 2024. Reasons: errors in the text; lack of ethics approval or compliance; a conflict of interest; concerns about the data.

### Direct molecular detection from clinical samples

qPCR on the *rpb1* gene was used to confirm the presence of *T*. *tenax* directly from clinical samples using specific primers and probe **(Fig 1E)**. Cross amplifications were prevented *in silico* and primers were tested on the DNA of *Trichomonas vaginalis* strain G3 (ATCCPRA-98). DNA extraction from our isolates and specimens were performed using the NucleoSpin Tissue kit (Macherey-Nagel, Hoerdt, France). The optimized 20 μL Quantitative Real-Time Polymerase Chain Reaction (qPCR) mix contained: master mix (10 μL), primers (0.5 μL, 20 nM), probe (0.5 μL, 5 nM), water (3.5 μL) and 5 μL of DNA. qPCR temperature cycle was: DNA activation at 50°C for two minutes, denaturation at 95°C for five minutes, followed by 40 cycles of 95°C for one second and 60°C for 30 seconds for the plate read. qPCR tubes were deposited in a CFX96 Touch thermal cycler (Bio-rad, France). The results were normalized by testing the gene encoding albumin in parallel. The primers used were: Forward: 5’- GCTGTCATCTCTTGTGGGCTG T-3’, Reverse: 5’- AAACTCATGGGAGCTGCTGGTTC-3’ and FAM probe: 6FAM- 5’ CCTGTCATGCCCACACAAATCTCTCC-3’[38]. A ratio of the cycle threshold (Ct) obtained in q-PCR for the *rpb1* gene and the albumin gene was calculated. (**S3 Table).**

### Statistical analysis

The statistical analysis was performed using “R” software (Version 3.5.1) using a ordinal logistic regression with a four-modalities qualitative variable to investigate the correlation between health status and detection methods (culture or PCR) with the existence of *T*. *tenax*.

χ^2^ tests for sex and smoking status descriptive statistics and Fisher test for the phylogenetic tree analysis using *Statistical Package for the Social Sciences* (SPSS Inc, IBM Company).

## Results

### Isolation of *Trichomonas* sp.

Fifty-three strains of *Trichomonas* sp. were obtained from periodontal samples, 37/106 from patients with periodontitis and 16/85 from control patients (p = 0.018) (**Table 2, Table 3**). Six isolates were lost before conservation. Protists were likely to be *T*. *tenax* based on their morphology as observed by microscopy. For a definitive identification, we first performed alignment of available *rpb1* gene using online Clustal Omega [39] with standard parameters for 11 sequences of *Trichomonas* spp. and we visualized it using MView online software (http://www.ebi.ac.uk/Tools/msa/mview/). Following the 100% consensus sequence available (**S1 Scheme**), we designed degenerated primers on conserved regions between the 11 different *Trichomonadidae* strains. In order to evaluate the intra-species diversity of the *rpb1* gene, we amplified and sequenced the *rpb1* gene from 15 randomly chosen strains isolated from our control and diseased patients. Of the 3,000 base pairs obtained, all sequences were 100% identical to the reference strain *T*. *tenax* NIH4, except one strain (number 13) which possesses two synonym single nucleotide polymorphisms (SNP). All remaining isolates were identified as *T*. *tenax* using our specific primers.

The article "Specific clones of Trichomonas tenax are associated with periodontitis" was retracted in 2024. Reasons: errors in the text; lack of ethics approval or compliance; a conflict of interest; concerns about the data.

**Table 2:** Frequency of *Trichomonas tenax* by qPCR and culture.

	Culture		qPCR		Culture or qPCR	
	Controls	Patients	Controls	Patients	Controls	Patients
**Negative**	69 (81,2%)	69 (65,1%)	61 (71,8%)	70 (66%)	61 (71.8%)	61(57.5%)
**Positive**	16 (18,2%)	37 (34,9%)	24 (28,2%)	36 (34%)	24 (28.2%)	45 (42.5%)
**Total**	85	106	85	106	85	106

**Table 3:** Comparison between frequency of qPCR and culture.

		Culture		
		Negative	Positive	Total
**Real-Time PCR**	**Negative**	122 (88,4%)	9 (17%)	131
	**Positive**	16 (11,6%)	44 (83%)	60
	**Total**	138	53	191

### Detection of *T*. *tenax* using quantitative real time PCR

Sixty of the 191 samples were positive for *T*. *tenax*, 24/85 controls and 36/106 periodontitis patients (p = 0.089) (**Table 2; Table 3**). The standardized results using the average ratio of the *rpb1* gene on the albumin gene demonstrate the absence of a link between the amount of *Trichomonas* DNA and the pathological status (p = 0.087, χ^2^) (**S3 Table**).

### Combined results

A good correlation was observed between qPCR and culture, as 83% of positive cultures were also positive for qPCR and 88% of negative cultures were also negative for qPCR. By combining both results, 45/106 patients were positive by culture and/or PCR, compared to 24/85 of controls (p = 0.042, χ^2^). No association could be found with the patient's gender and health status (p = 0.710, χ2) or with the detection of *T*. *tenax* (p = 0.485, χ^2^). The carriage of *T*. *tenax* and smoking status are correlated regardless of health status (p = 0.001, χ^2^). Regarding the periodontitis classification of each patient, *T*. *tenax* is significantly more detected in severe periodontitis than in mild or moderate periodontitis (p<0.05).

The article "Specific clones of Trichomonas tenax are associated with periodontitis" was retracted in 2024. Reasons: errors in the text; lack of ethics approval or compliance; a conflict of interest; concerns about the data.

### Genome sequencing

The 46,742,176 base pair (bp) draft genome obtained contains 4,161 scaffolds with a N50 of 13,554 bp with a minimum of 4,002 bp to a maximum of 92,188 bp with a G+C content estimated of about 34.6% similar to *T*. *vaginalis* G3 (35.5%). The gene prediction determined 34,291 Open Reading Frame (ORF) includes 21,854 proteins that could be annotated and 12,437 ORFans. Of these, 21,193 proteins are in common with *T*. *vaginalis*, and only five with *Trichomonas gallinae*, four with *T*. *tenax* (sequences of the same strain already available on the nr database) and one with *Tritrichomonas foetus*. This high number of best hits shared with *T*. *vaginalis* G3 strain is logical, as this species in the only species of *Trichomonas* spp. for which a draft genome is available. In the *T*. *vaginalis* G3 genome, about 250 genes were annotated as ribosomal proteins [40]. In *T*. *tenax*, we obtained in the draft 52 ORFs annotated as the 40S ribosome and 68 annotated as the 60S ribosome. We isolated the complete sequence of the *rpb1* gene measuring 4,962 nucleotides and, congruently, the alignment with the same strain in the database showed 61% of coverage with 100% identity. The alignment starts at position 229 and finishes at position 3,276 of the complete sequence and makes the 3’end of this gene available.

### MLST typing

Four housekeeping genes were extracted based on the *T*. *vaginalis* typing system: Alanyl tRNA synthetase (ALTS), DNA mismatch repair protein (DMRP), Serine hydromethyltransferase (SHMT), and Mannose-6-phosphate isomerase (M6PI). For genes for which no homologs of *Trichomonas vaginalis* could be detected in our *T*.*tenax* draft genome, we chose three genes because of their functional similarity to complete the system: Glutamine amidotransferase class-I (GAT1), Histidyl tRNA synthetase (HIST), Cysteinyl tRNA synthetase (CYST) (**Table 1**). The 47 strains and the reference NIH4 strain are clustered into three major groups: strains obtained in the control group are significantly predominant in group 1 and strains isolated in periodontitis patients are significantly predominant in group 3 (p <0.05, Fisher). Only periodontal patient strains constitute the cluster 2. (**Fig 2**). Phylogenetic tree analysis, based on each housekeeping gene, showed similar topologies. Indeed, six of seven genes also present three major clusters, namely the DMRP, SHMT, ALTS, SHMT, M6PI and GAT1 gene (**S1–S7 Figs**). Concerning the tree based on the CYST gene, all sequences are identical between controls and patients, highlighting the conservation and lack of variability in this portion of the gene. All strain sequences obtained for each gene portion were compared with the sequences of the reference strain *T*. *tenax* NIH4 to investigate the presence of a single nucleotide polymorphism (SNP) (**S2 Table**). Four isolates had the same genotype, while the others 43 isolates each had a specific genotype.

The article "Specific clones of Trichomonas tenax are associated with periodontitis" was retracted in 2024. Reasons: errors in the text; lack of ethics approval or compliance; a conflict of interest; concerns about the data.

**Fig 2:** *Trichomonas tenax* relationship based on multilocus sequence typing phylogenetic analysis. Maximum likelihood phylogenetic tree of *T*. *tenax* strains. Colors legend: black for patients, blue for control and red for reference strain.

## Discussion

In this study, by combining a polyphasic approach that associates culture and qPCR, we found a correlation between periodontitis and the presence of *T*. *tenax* (p< 0.05). Although *T*. *tenax* is more frequently detected by qPCR in patients than in controls, the difference is not significant (p = 0.435). A significant difference was observed using culture only (p = 0.015). By combining the culture and PCR results to neutralize the effect of false negative of each technique and evaluate the real prevalence of *T*. *tenax*, the difference is significant (p = 0.042). The probability of false positive/negative frequency is reduced due to the good correlation observed between both techniques: 83% of positive cultures also positive for qPCR and 88% of negative cultures also negative for q-PCR techniques. We believe that this good correlation indicates that the culture and handling protocols, including the transport medium specifically developed for anaerobic microorganisms, were highly efficient. However, as commonly observed in clinical microbiology, the higher sensitivity of the PCR suggests that some *T*. *tenax* did not grew in culture. The reasons are unknown but usually because microorganisms are dead at time of inoculation due to delayed inoculation between sampling and culture, quality of the operator or quality of the batch of transport or culture media. The 11.6% of the positive samples in culture not identified by real-time PCR shows that false positive occur also with molecular amplification, usually as a consequence of inhibitors.

Furthermore, positive culture in controls underlines the difficulty of having a true negative control group. We first suspected that a higher rate of positive culture in periodontitis patients could have been the result of a higher concentration of protist in these samples. But the absence of such differences observed using quantitative PCR disproves this hypothesizes. Indeed, no difference in the amount of *T*. *tenax* DNA in controls and patients is demonstrated after normalization of the results by the albumin gene. A recent review reports higher prevalence of *T*. *tenax* occurrence in gum diseased (gingivitis and periodontitis) in most studies present in the literature and explains that the heterogeneity of the prevalence observed may be due to the different methods used to detect the protist (majority of microscopic observation, insufficient use of molecular biology) and the studied population diversity [21]. The same limits may be pointed out in another study reporting the absence of trichomonas in healthy sites in periodontitis patients [27]. Theses discrepancies, as compared to our study, could be related with false positive of our PCR procedure. However, the high level of positive culture herein is not in agreement with this hypothesis and the detection of trichomonads from healthy sites in controls with no periodontal disease indicated that *T*. *tenax* carriage remains common in the oral cavity.

The article "Specific clones of Trichomonas tenax are associated with periodontitis" was retracted in 2024. Reasons: errors in the text; lack of ethics approval or compliance; a conflict of interest; concerns about the data.

A correlation could also be established between the severity of periodontitis and the presence of protists (p<0.05). *T*. *tenax* is found in severe periodontitis differing from other periodontitis, by the depth of the pocket as well as the loss of attachment. The environment of severe periodontitis would therefore be more favorable to the development of the protist and other bacteria species leading to serious lesions and inflammatory responses.

We now suspect that the specific periodontal microbiota associated with periodontitis could promote the growth of *T*. *tenax*. Indeed, when inoculated in the culture medium, the sample also contains bacterial microbiota of dental pockets. Indeed, periodontitis is suspected to be due to an inflammatory response to microorganisms [1,8]. Finally, no single microorganism is implicated but rather a combination of microorganisms act synergistically [3,17,20]. Investigating the difference in microbiota between healthy individuals and patients with mild and moderate periodontitis compared to severe periodontitis would highlight the combined role of protist and oral microbiome.

Several studies have demonstrated the efficacy of PCR in detecting *T*. *tenax* by employing rRNA sequencing [41]. Likewise, oral cavity metagenomics studies have identified significant *T*. *tenax* rRNA intergenic spacers [42]. Nonetheless, these systems come up against identification limits. Designing primers based on the *rpb1* gene according to Malik *et al*. [33], allowed us to create a highly specific and sensitive system: this gene is both discriminatory between different species and genotypes and is highly conserved within the same species [43,44]. All isolated strains of *Trichomonas sp*. were identified as *T*. *tenax*, once again demonstrating the effectiveness of this primer system and the extreme conservation of *T*. *tenax* based on the *rpb1* gene.

The article "Specific clones of Trichomonas tenax are associated with periodontitis" was retracted in 2024. Reasons: errors in the text; lack of ethics approval or compliance; a conflict of interest; concerns about the data.

Finally, the MLST system made it possible to investigate the clonal relationship between the protist and periodontitis based on the system created for the closely studied neighboring species, *T*. *vaginalis* [35]. The data obtained reveal the existence of three clusters grouping *T*. *tenax*, suggesting genetically diverse strains affecting the periodontium tissue. A significant association could be observed between clustering and the occurrence of periodontitis. The possibility of finding new virulence factors in common between strains in future work could confirm the virulence of diseased strains related to the severity of the periodontal disease. Recently, a physiopathology mechanism of *T*. *tenax* has been described in the periodontitis disease: *T*. *tenax* induced an effect against the human macrophage and deregulates the proinflammatory cytokines [45]. Furthermore, *in vitro* studies showed that *T*. *tenax* had cytotoxic effects on mammalian cells [46]. An animal model reproducing periodontitis suggested in these recent studies could be used to explore the potential pathophysiological role of *T*. *tenax* [21,47].

## Conclusion

A high prevalence of *T*. *tenax* in both controls and patients is detected using genomic-dependent and culture-based methods of detection. *T*. *tenax* was more frequently associated with severe periodontitis. Three clusters of strains were highlighted by the MLST genotyping system, two were significantly associated with periodontitis. *T*. *tenax* appears to be associated with the onset or/and evolution of periodontal diseases. However, although these differences are statistically significant, it is impossible to determine whether they are a cause or a consequence of the disease.

## Supporting information

S1 Scheme Quantitative Real-Time PCR (q-RT PCR) specific for *Trichomonas tenax*. (DOCX)

S1 Table The table below presents the classification of each patient. The numbers correspond to a patient and preserve anonymity. The discontinuity of the numbering is linked to the change of operator in the laboratory. In black: patients with periodontitis.—In bold: the patient controls.
(DOCX)

S2 Table Sequence types of *Trichomonas tenax* based on single-nucleotide polymorphism against the *Trichomonas tenax* reference strain. In bold: the number of sequences types.
(DOCX)

S3 Table The table below presents the cycle threshold obtained in q-PCR for the *RPB1*gene and the albumin gene for the standardization. In black: periodontitis patients. In bold: controls.
(DOCX)

S1 Fig *Trichomonas tenax* phylogenetic analysis based on Alanyl tRNA synthetase (ALTS) gene. In black: patients with periodontitis. In blue: the patient controls.
(TIFF)

S2 Fig *Trichomonas tenax* phylogenetic analysis based on DNA mismatch repair protein (DMRP) gene. In black: patients with periodontitis. In blue: the patient controls.
(TIFF)

S3 Fig *Trichomonas tenax* phylogenetic analysis based on Serine hydromethyltransferase (SHMT) gene. In black: patients with periodontitis. In blue: the patient controls.
(TIFF)

S4 Fig *Trichomonas tenax* phylogenetic analysis based on Mannose -6-phosphate isomerase (M6PI) gene. In black: patients with periodontitis. In blue: the patient controls.
(TIFF)

S5 Fig *Trichomonas tenax* phylogenetic analysis based on Glutamine amidotransferase class-I (GAT1) gene. In black: patients with periodontitis. In blue: the patient controls.
(TIFF)

S6 Fig *Trichomonas tenax* phylogenetic analysis based on Histidyl tRNA synthetase (HIST) gene. In black: patients with periodontitis. In blue: the patient controls.
(TIFF)

S7 Fig *Trichomonas tenax* phylogenetic analysis based on Cysteinyl tRNA synthetase (CYST) gene. In black: patients with periodontitis. In blue: the patient controls.
(TIFF)

The article "Specific clones of Trichomonas tenax are associated with periodontitis" was retracted in 2024. Reasons: errors in the text; lack of ethics approval or compliance; a conflict of interest; concerns about the data.

## References

[1] PihlstromBL, MichalowiczBS, JohnsonNW. Periodontal diseases. Lancet (London, England). 2005;366: 1809–20. 10.1016/S0140-6736(05)67728-816298220

[2] TonettiMS, GreenwellH, KornmanKS. Staging and grading of periodontitis: Framework and proposal of a new classification and case definition. J Clin Periodontol. 2018;45: S149–S161. 10.1111/jcpe.12945 29926495

[3] SocranskySS, Haffajee aD, CuginiM a, SmithC, KentRL. Microbial complexes in subgingival plaque. J Clin Periodontol. 1998;25: 134–144. 10.1111/j.1600-051X.1998.tb02419.x 9495612

[4] RosierBT, De JagerM, ZauraE, KromBP. Historical and contemporary hypotheses on the development of oral diseases: are we there yet? Front Cell Infect Microbiol. 2014; 10.3389/fcimb.2014.00092 25077073PMC4100321

[5] AssumaR, OatesT, CochranD, AmarS, GravesDT. IL-1 and TNF antagonists inhibit the inflammatory response and bone loss in experimental periodontitis. J Immunol. 1998;160: 403–9. 9551997

[6] NocitiFH, CasatiMZ, DuartePM. Current perspective of the impact of smoking on the progression and treatment of periodontitis. Periodontol 2000. 2015;67: 187–210. 10.1111/prd.12063 25494601

[7] LallaE, PapapanouPN. Diabetes mellitus and periodontitis: a tale of two common interrelated diseases. Nat Rev Endocrinol. 2011;7: 738–48. 10.1038/nrendo.2011.106 21709707

[8] KinaneDF, StathopoulouPG, PapapanouPN. Periodontal diseases. Nat Rev Dis Prim. Macmillan Publishers Limited; 2017;3: 17038 10.1038/nrdp.2017.38 28805207

[9] GeX, RodriguezR, TrinhM, GunsolleyJ, XuP. Oral microbiome of deep and shallow dental pockets in chronic periodontitis. PLoS One. Public Library of Science; 2013;8: e65520 10.1371/journal.pone.0065520 23762384PMC3675156

The article "Specific clones of Trichomonas tenax are associated with periodontitis" was retracted in 2024. Reasons: errors in the text; lack of ethics approval or compliance; a conflict of interest; concerns about the data.

[10] WangJ, QiJ, ZhaoH, HeS, ZhangY, WeiS, et al Metagenomic sequencing reveals microbiota and its functional potential associated with periodontal disease. Sci Rep. Nature Publishing Group; 2013;3: 1843 10.1038/srep01843 23673380PMC3654486

[11] GriffenAL, BeallCJ, CampbellJH, FirestoneND, KumarPS, YangZK, et al Distinct and complex bacterial profiles in human periodontitis and health revealed by 16S pyrosequencing. ISME J. Nature Publishing Group; 2012;6: 1176–85. 10.1038/ismej.2011.191 22170420PMC3358035

[12] GalimanasV, HallMW, SinghN, LynchMD, GoldbergM, TenenbaumH, et al Bacterial community composition of chronic periodontitis and novel oral sampling sites for detecting disease indicators. Microbiome. 2014;2 10.1186/2049-2618-2-32 25225610PMC4164120

[13] KumarPS, GriffenAL, BartonJA, PasterBJ, MoeschbergerML, LeysEJ. New bacterial species associated with chronic periodontitis. J Dent Res. 2003;82: 338–344. 10.1177/154405910308200503 12709498

[14] BikEM, LongCD, ArmitageGC, LoomerP, EmmersonJ, MongodinEF, et al Bacterial diversity in the oral cavity of ten healthy individuals. Isme J. 2010;4: 962–974. 10.1038/ismej.2010.30 20336157PMC2941673

[15] LyM, AbelesSR, BoehmTK, Robles-SikisakaR, NaiduM, Santiago-RodriguezT, et al Altered Oral Viral Ecology in Association with Periodontal Disease. MBio. 2014;5: e01133-14–e01133-14. 10.1128/mBio.01133-14 24846382PMC4030452

[16] Duran-PinedoAE, ChenT, TelesR, StarrJR, WangX, KrishnanK, et al Community-wide transcriptome of the oral microbiome in subjects with and without periodontitis. ISME J. Nature Publishing Group; 2014;8: 1659–72. 10.1038/ismej.2014.23 24599074PMC4817619

[17] CappuynsI, GugerliP, MombelliA. Viruses in periodontal disease—a review. Oral Dis. Munksgaard International Publishers; 2005;11: 219–229. 10.1111/j.1601-0825.2005.01123.x 15984953

[18] HershSM. Pulmonary trichomoniasis and Trichomonas tenax. J Med Microbiol. 1985;20: 1–10. 10.1099/00222615-20-1-1 3894667

[19] LyonsT, ScholtenT, PalmerJC, StanfieldE. Oral amoebiasis: the role of Entamoeba gingivalis in periodontal disease. Quintessence Int Dent Dig. 1983;14: 1245–1248. 6585855

[20] BonnerM, AmardV, Bar-PinatelC, CharpentierF, ChatardJ-M, DesmuyckY, et al Detection of the amoeba Entamoeba gingivalis in periodontal pockets. Parasite. 2014;21: 30 10.1051/parasite/2014029 24983705PMC4077299

[21] MartyM, LemaitreM, KémounP, MorrierJ, MonsarratP. Trichomonas tenax and periodontal diseases: a concise review. 2017; 10.1017/S0031182017000701 28583214

The article "Specific clones of Trichomonas tenax are associated with periodontitis" was retracted in 2024. Reasons: errors in the text; lack of ethics approval or compliance; a conflict of interest; concerns about the data.

[22] CanabarroA, ValleC, FariasMR, SantosFB, LazeraM, WankeB. Association of subgingival colonization of Candida albicans and other yeasts with severity of chronic periodontitis. J Periodontal Res. 2013;48: 428–32. 10.1111/jre.12022 23137301

[23] CepickaI, HamplV, KuldaJ. Critical Taxonomic Revision of Parabasalids with Description of one New Genus and three New Species. Protist. 2010;161: 400–433. 10.1016/j.protis.2009.11.005 20093080

[24] BrookB, SchusterFL. Oral Protozoa: Survey, Isolation, and Ultrastructure of Trichomonas tenax from Clinical source. Trans Am Microsc Soc. 1984;103: 376–382.

[25] MaritzJM, LandKM, CarltonJM, HirtRP. What is the importance of zoonotic trichomonads for human health? Trends Parasitol. Elsevier Ltd; 2014;30: 333–341. 10.1016/j.pt.2014.05.005 24951156PMC7106558

[26] GhabanchiJ, ZibaeiM, AfkarMD, SarbazieAH. Prevalence of oral Entamoeba gingivalis and Trichomonas tenax in patients with periodontal disease and healthy population in Shiraz, southern Iran. Indian J Dent Res. 2010;21: 89–91. 10.4103/0970-9290.62821 20427914

[27] BissonC, LecP-H, BliqueM, ThillyN, MachouartM. Presence of trichomonads in subgingival biofilm of patients with periodontitis: preliminary results. Parasitol Res. 2018; 10.1007/s00436-018-6077-2 30215136

[28] DuboucherC, MogenetM, PériéG. Salivary trichomoniasis. A case report of infestation of a submaxillary gland by Trichomonas tenax. Arch Pathol Lab Med. 1995;119: 277–9. 7887784

[29] DuboucherC, Farto-BensassonF, ChéronM, PeltierJY, BeaufilsF, PériéG. Lymph node infection by Trichomonas tenax: report of a case with co-infection by Mycobacterium tuberculosis. Hum Pathol. 2000;31: 1317–21. 10.1053/hupa.2000.18502 11070125

[30] LewisKL, DohertyDE, RibesJ, SeaboltJP, BensadounES. Empyema caused by trichomonas. Chest. 2003;123: 291–2. 1252763510.1378/chest.123.1.291

[31] MehrAK, ZarandiA, AnushK. Prevalence of Oral Trichomonas tenax in Periodontal Lesions of Down Syndrome in Tabriz, Iran. J Clin Diagn Res. 2015;9: ZC88–90. 10.7860/JCDR/2015/14725.6238 26393213PMC4573046

[32] EkePI, PageRC, WeiL, Thornton-EvansG, GencoRJ. Update of the Case Definitions for Population-Based Surveillance of Periodontitis. J Periodontol. 2012;83: 1449–1454. 10.1902/jop.2012.110664 22420873PMC6005373

[33] MalikSB, BrochuCD, BilicI, YuanJ, HessM, LogsdonJM, et al Phylogeny of parasitic parabasalia and free-living relatives inferred from conventional markers vs. Rpb1, a single-copy gene. PLoS One. 2011;6 10.1371/journal.pone.0020774 21695260PMC3111441

[34] HyattD, ChenG-L, LocascioPF, LandML, LarimerFW, HauserLJ. Prodigal: prokaryotic gene recognition and translation initiation site identification. BMC Bioinformatics. 2010;11: 119 10.1186/1471-2105-11-119 20211023PMC2848648

The article "Specific clones of Trichomonas tenax are associated with periodontitis" was retracted in 2024. Reasons: errors in the text; lack of ethics approval or compliance; a conflict of interest; concerns about the data.

[35] CorneliusDC, RobinsonDA, MuznyCA, MenaLA, AanensenDM, LushbaughWB, et al Genetic characterization of Trichomonas vaginalis isolates by use of multilocus sequence typing. J Clin Microbiol. 2012;50: 3293–3300. 10.1128/JCM.00643-12 22855512PMC3457461

[36] BenamarS, CassirN, MerhejV, JardotP, RobertC, RaoultD, et al Multi-spacer typing as an effective method to distinguish the clonal lineage of Clostridium butyricum strains isolated from stool samples during a series of necrotizing enterocolitis cases. J Hosp Infect. 2017;95: 300–305. 10.1016/j.jhin.2016.10.026 27988045

[37] PriceMN, DehalPS, ArkinAP. Fasttree: Computing large minimum evolution trees with profiles instead of a distance matrix. Mol Biol Evol. 2009;26: 1641–1650. 10.1093/molbev/msp077 19377059PMC2693737

[38] CarcopinoX, HenryM, BenmouraD, FallabreguesAS, RichetH, BoubliL, et al Determination of HPV type 16 and 18 viral load in cervical smears of women referred to colposcopy. J Med Virol. 2006;78: 1131–40. 10.1002/jmv.20673 16789021

[39] SieversF, WilmA, DineenD, GibsonTJ, KarplusK, LiW, et al Fast, scalable generation of high-quality protein multiple sequence alignments using Clustal Omega. Mol Syst Biol. 2011;7: 539 10.1038/msb.2011.75 21988835PMC3261699

[40] CarltonJM, HirtRP, SilvaJC, DelcherAL, SchatzM, ZhaoQ, et al Draft Genome Sequence of the Sexually Transmitted Pathogen Trichomonas vaginalis. Alias J Smith Terry R Utterback Kazutoyo Osoegawa Pieter J Jong John M Logsdon Jr Sci. 2007;11: 207–212.10.1126/science.1132894PMC208065917218520

[41] MallatH, PodglajenI, LavardeV, MainardiJ, FrappierJ, CornetM. Molecular Characterization of Trichomonas tenax Causing Pulmonary Infection. 2004;42: 3886–3888. 10.1128/JCM.42.8.3886PMC49758915297557

[42] Belda-FerreP, AlcarazLD, Cabrera-RubioR, RomeroH, Simón-SoroA, PignatelliM, et al The oral metagenome in health and disease. ISME J. Nature Publishing Group; 2012;6: 46–56. 10.1038/ismej.2011.85 21716308PMC3246241

[43] BilicI, JaskulskaB, SouillardR, LiebhartD, HessM. Multi-Locus Typing of Histomonas meleagridis Isolates Demonstrates the Existence of Two Different Genotypes. Leung FCC, editor. PLoS One. Public Library of Science; 2014;9: e92438 10.1371/journal.pone.0092438 24658534PMC3962415

[44] HussainI, JaskulskaB, HessM, BilicI. Detection and quantification of Histomonas meleagridis by real-time PCR targeting single copy genes. Vet Parasitol. 2015;212: 382–388. 10.1016/j.vetpar.2015.08.011 26319200

[45] GovroEJ, StuartMK. Cytokine response of human THP-1 macrophages to Trichomonas tenax. Exp Parasitol. 2016;169: 77–80. 10.1016/j.exppara.2016.07.011 27497807

The article "Specific clones of Trichomonas tenax are associated with periodontitis" was retracted in 2024. Reasons: errors in the text; lack of ethics approval or compliance; a conflict of interest; concerns about the data.

[46] RibeiroLC, SantosC, BenchimolM. Is Trichomonas tenax a Parasite or a Commensal? Protist. Elsevier GmbH.; 2015;166: 196–210. 10.1016/j.protis.2015.02.002 25835639

[47] LemaitreM, MonsarratP, Blasco-BaqueV, LoubièresP, BurcelinR, CasteillaL, et al Periodontal Tissue Regeneration Using Syngeneic Adipose-Derived Stromal Cells in a Mouse Model. Stem Cells Transl Med. 2017;6: 656–665. 10.5966/sctm.2016-0028 28191762PMC5442818

